# Transversus Abdominis Plane Block Versus Local Anesthetic Wound Infiltration for Postoperative Analgesia in Adult Patients Undergoing Hernia Repair in Daycare Procedure: A Randomized Control Trial

**DOI:** 10.7759/cureus.21311

**Published:** 2022-01-17

**Authors:** Sidra Mukhtar, Madeha Ishag Adam, Estefania Martinez-Jimenez, Hamza Naseem, Insiya Sherawala, Shivani M Mehta, Fares Mohammed Saeed Muthanna, Abdul Muqtadir, Rahil Barkat

**Affiliations:** 1 Internal Medicine, Mayo Hospital, Karachi, PAK; 2 Neurogenerative Disease, Fujian Medical University, Fuzhou, CHN; 3 Medical School, Universidad Autonoma del Estado de Hidalgo, Pachuca, MEX; 4 Medical School, Jinnah Medical and Dental College, Karachi, PAK; 5 Medical School, Bharati Vidyapeeth Deemed Medical College, Pune, IND; 6 Medical School, Xavier University School of Medicine, Oranjestad, ABW; 7 Department of Pharmacy, Walailak University, Nakhon Si Thammarat, THA; 8 Medicine and Surgery, Shadan Institute of Medical Sciences, Dr. NTR University of Health Sciences, Hyderabad, IND; 9 Indus Hospital Research Center, The Indus Hospital, Karachi, PAK

**Keywords:** postoperative, analgesia, hernia repair, local anesthetic wound infiltration, transversus abdominis plane block

## Abstract

Introduction: Various modalities are now being used to manage postoperative pain, such as regional nerve blocks techniques, continuous epidural analgesia, patient-controlled analgesia, opioids, and systemic non-steroidal anti-inflammatory drugs. This study compared the mean postoperative pain score between ultrasound-guided transversus abdominis plane (TAP) block and a local anesthetic wound infiltration at the surgical incision site.

Methodology: A prospective, comparative, randomized controlled trial (RCT) was carried out from February 2021 to September 2021. The study was conducted in the anesthesia department of Dow University of Health Sciences, Karachi, Pakistan. Patients aged 18-80 years presenting with elective surgery of (both direct and indirect) inguinal hernia repair were enrolled in the study. Participants were randomly assigned into one of the two groups that are local anesthetic wound infiltration (Group A) and TAP block (Group B). The mean pain score was assessed using a visual analog scale and compared between the two groups.

Results: The study included 168 patients grouped in two different groups. The mean age in Group A was 43.87 (+17.21), and Group B was 47.01 (±15.37). Mean pain scores in groups A and B were 6.36±1.94 vs 4.51 ± 1.99 (p-value=0.001). The pain rescue medications were given to 57.14% of patients in Group A and 34.52% of patients in Group B, and it was significantly different in the two groups (p-value=0.003). It was found that patients in Group A reported more severe pain (41.67%) than patients in Group B (10.71%).

Conclusion: When compared to local anesthetic wound infiltration, ultrasound-guided TAP block had better analgesic activity compared to local anesthetic wound infiltration.

## Introduction

Acute postoperative pain is a prevalent condition that pain specialists and all healthcare practitioners face daily [1]. Pain management is an essential part of perioperative anesthetic care. However, the impact of initial postoperative pain control on surgical outcomes is debatable [2]. It is believed that pain is one of the primary reasons for a prolonged hospital stay, patient dissatisfaction, and primary care consultation [3].

Various modalities are now being used to manage postoperative pain, such as regional nerve blocks techniques, continuous epidural analgesia, patient-controlled analgesia, opioids, and systemic non-steroidal anti-inflammatory drugs [4]. One of the most commonly used modalities for postoperative pain management is local anesthetic infiltration at the surgery site [5]. Transversus abdominis plane (TAP) block is a regional anesthesia technique in which neural afferents to the anterior abdominal wall’s parietal peritoneum, skin, and muscles are blocked to provide analgesia [6]. It blocks T6-L1 lower or mid thoracic and upper lumbar spinal nerves. It is indicated in different surgical procedures to provide analgesia [7].

Traditional local anesthetic wound infiltration (WI) is another method in which local anesthesia is injected into the surgery site. Surgeons also favor it because of its convenience, and it is utilized for postoperative analgesia in many regions [8]. However, a newer technique, TAP block, is becoming increasingly popular among anesthetists as a mode of postoperative analgesia in patients undergoing hernia repair. However, even though earlier studies favoring analgesic efficacy of TAP block over infiltration of wound with local anesthetic, more recent studies have yielded contradictory results, rending the superiority of TAP block still questionable [6]. The outcome of this study will either help us adapt to the newer technique (TAP block), if found to be more effective, or if not, it will guide us to continue to the conventional technique of infiltration of a wound with local anesthetics.

Many clinicians have recently begun to utilize TAP block and compare it to WI to decide which block is better in adults because of the significant advancement of ultrasound methods; nonetheless, the results are still ambiguous. Thus, the study compares the mean postoperative pain score between ultrasound-guided TAP block and a local anesthetic drug’s WI at the surgical incision site.

## Materials and methods

Methodology

It was a prospective, comparative, randomized controlled trial (RCT) from February 2021 to September 2021. The study was conducted in the anesthesia department at the Dow University of Health Sciences, Karachi, Pakistan. After getting ethical approval from the Institutional Review Board (IRB) of Dow University of Health Sciences, the study was conducted.

Sample size and sampling technique

The same size was calculated using OpenEpi by considering absolute population proportion in groups A and B as 0.55 and 0.33, respectively [4], 95% CI, 80% power, and absolute precision of 0.05. The calculated sample size (n) was 84 in each group.

Eligibility criteria

The inclusion criteria included patients aged 18-80 years presenting with elective surgery of (both direct and indirect) inguinal hernia repair under general anesthesia with the endotracheal intubation. The exclusion criteria were body mass index > 35 kg/m^2^, existing neurologic disease, ASA (American Society of Anesthesiologists) grade ≥III patients, previous history of abdominal surgeries, and patients having a history of hypersensitivity of local anesthesia agents.

Intervention

After identifying eligible patients, written consent was taken from them. Participants were randomized in a parallel design with a computer-generated assignment to either local anesthetic WI group (Group A) and TAP block (Group B) in a 1:1 ratio. Study drugs were prepared in the hospital pharmacy by trained pharmacists. It was placed in envelopes containing medications for groups A or B. The envelopes were sealed, and the name of the project and consecutive numbers were marked as per a computer-generated block randomization list prepared by the hospital pharmacy. Boxes were opened, and syringes were filled by operation theater nurses who were not a part of the study and postoperative care of patients.

Intravenous access was obtained inside the operation room and a monitor was attached. Baseline blood pressure, heart rate, and respiratory rate were obtained. Induction was done utilizing injection. Midazolam 0.02 mg/kg, while inj. fentanyl 3 μg/kg and propofol 2 mg/kg were used for analgesia. Anesthesia was maintained by a 50:50 mixture of air and oxygen, as well as 1-1.5% of isoflurane.

Patients in Group A were provided with local anesthetic infiltration at a surgical wound site at the end of surgery. The anesthesiologist provided 10 ml of 0.25% bupivacaine through an aseptic method to the operating surgeon, who deposited 5 ml of bupivacaine above and 5 ml of bupivacaine below the surgical incision site.

Group B patients received ultrasound-guided TAP block after surgery with 10 ml of 0.25% bupivacaine. Patients were lying in a supine position and TAP block was performed unilaterally using ultrasound guidance and placed in a transverse plane perpendicular to the line joining the iliac crest and the inferior rib on the anterolateral part of the abdominal wall between the iliac crest and costal margin. A transverse view of abdominal muscle layers was obtained, and subcutaneous tissue, external oblique muscle, internal oblique muscle, and transversus-abdominis muscle were identified, superficial to deep, respectively. The fascia was recognized between the internal oblique muscle and transversus-abdominis muscle. As a block needle, a 22 G spinal needle was used, which was inserted anteriorly through an in-plane approach and advanced under ultrasound observation. The drug was injected, and the placement was confirmed by hypoechoic injectate deposition and hydrodissection of the TAP.

Outcome measures

All the patients who recovered from general anesthesia and pain were assessed at 2, 4, and 6 hours. Postoperative pain was assessed using a visual analog scale (VAS) ranging from 0 to 10, on which 0 means no pain and 10 showed worst pain. A higher score indicates the worst outcome. A score of 0 was taken as no pain, a score of 1-3 was considered mild pain, 3-6 was considered moderate pain, and 7-10 as severe pain. The nurse assessed the outcome, and both the nurse and patients were blinded and unaware about the group they were in to prevent any bias in the study. Secondary outcomes included a number of patients requesting pain-relief medications and the mean time to first pain-relief medication.

For pain-relief medications, intravenous morphine was provided to the patient on request for the first 2 hours in the postoperative care unit. The initial dose of morphine was 5 mg, with subsequent doses of 2.5 mg and a minimum of 10 minutes between them. From 2 to 6 hours postoperatively, oral ketobemidone 2.5 mg was given based on the patient’s decision. For nausea complain, ondansetron was administered with the first dose of 4 mg followed by 1 mg if required. No prophylactic antiemetics were administered.

Statistical analysis

For data analysis, STATA version 16.0 (StataCorp, College Station, TX, USA) was used. Normality of mean pain score and mean time to first pain-relief medication was assessed using Shapiro-Wilk test. Both followed the normal distribution. Mean and standard deviation were reported for continuous variables including mean pain score and mean time to first pain-relief medication, while frequency and percentages were reported for categorical variables. Characteristics of the two groups were compared using impendent t-test and chi-square independence test for continuous and categorical variables, respectively. A p-value less than 0.05 was considered significant.

## Results

The study included a total of 168 patients grouped in two different groups. The mean age in Group A was 43.87 (+17.21) and Group B was 47.01 (+15.37). There was no statistically significant difference in the age of the patients of both groups (p-value=0.134). The study had enrolled patients only of ASA I and II grades, and ASA grades of patients were significantly different in two groups (p-value=0.006). Patients’ weights were not significantly different in the two groups (p-value=0.861) as shown in Table 1.

**Table 1:** Comparison of baseline characteristics between study participants *Significant at p-value<0.05 ^Mean (standard deviation) SBP: systolic blood pressure; DBP: diastolic blood pressure

Variable	Group A	Group B	P-value
Age^	43.87 +/- 17.21	47.01 +/- 15.37	0.134
ASA grade n (%)			0.006*
I	63 (75.00)	46 (54.76)	
II	21 (25.00)	38 (45.24)	
Weight (kg)^	61.93 +/- 11.00	61.95 +/- 9.59	0.861
Preoperative vital signs			
Heart rate (beats/min)^	82.63 +/- 11.77	76.25 +/- 10.12	0.002*
Respiratory rate (breathe/min)^	17.41 +/- 2.39	17.11 +/- 2.24	0.406
SBP (mmHg)^	136.18 +/- 19.37	134.28 +/- 18.41	0.517
DBP (mmHg)^	78.57 +/- 11.14	81.73 +/- 7.80	0.034*

Mean pain scores in groups A and B were 6.36+1.94 and 4.51 ± 1.99, respectively (p-value=0.001). The pain-relief medication was given to 57.14% of patients in Group A and 34.52% of patients in Group B, and it was significantly different in the two groups (p-value=0.003). The mean time to the first pain-relief medication requirement was significantly lower in Group A (2.65+1.51) than in Group B (5.33+2.17) as the p-value was less than 0.05. As shown in Table 2, no significant difference was reported between the two groups in the incidence of nausea and vomiting. No reported cases of bruising, swelling, or bleeding at the TAP block injection site were recorded.

**Table 2:** Comparison of outcomes between two groups *Significant at p-value<0.05 ^Mean (standard deviation)

	Group A n(%)	Group B n(%)	P-value
Mean pain score^			
2 hours	3.71 +/- 1.09	3.22 +/- 1.26	0.266
4 hours	5.88 +/- 1.62	3.76 +/- 1.18	0.001*
6 hours	6.36 +/- 1.94	4.51 +/- 1.99	0.001*
Medication given for pain			
No	36 (42.86)	55 (65.48)	0.003*
Yes	48 (57.14)	29 (34.52)	
Mean time to first pain-relief medication (hours)^	2.65 +/- 1.51	5.33 +/- 2.17	0.001*
Nausea	38 (45.24)	35 (41.67)	0.255
Vomiting	36 (42.86)	33 (39.28)	0.361

## Discussion

One of the key concerns of both surgeons and their patients is postoperative pain control. Several methods have been used to achieve pain-free recovery of patients after surgery, such as peripheral nerve block, epidural analgesia, TAP block, and WI. TAP block can be performed using a landmark-based approach or under ultrasound guidance, and nowadays, it is commonly used in different surgical procedures. However, the current study has determined whether this technique is effective enough among patients who undergo lower abdominal surgery. Meanwhile, WI is a simple postoperative analgesic technique that has been frequently used. As a result, determining which technique is more effective in controlling postoperative pain would be beneficial.

The current study was conducted to compare the efficacy of TAP and local anesthetic WI in controlling pain among adult patients undergoing hernia repair in daycare procedures. In the current study, TAP block proved to be a better quality of analgesia than local anesthetic infiltration of surgical incision with less postoperative analgesic requirements. TAP block is efficient in patients undergoing abdominal surgeries like appendicectomy, open prostatectomy, cesarean section, abdominal hysterectomy, and laparoscopic cholecystectomy [9-11]. TAP block under ultrasound guidance was likewise proven to be simple, reliable, and safe. It was also discovered that while TAP block effects such as liver damage and intestinal hematoma are conceivable, they are less common with ultrasound guidance [12].

In the current study, pain relief concerning VAS and the requirement of pain-relief medication was assessed in both groups. Mean pain scores were significantly different in Group B than in local anesthetic WI. Our findings are consistent with those of other research regarding analgesia and postoperative opiate demand. Past studies have also shown that side effects are lower in Group B that can jeopardize the recovery of patients [13-14].

Decreasing postoperative requirements of morphine and associated side effects are desirable as these are vital to the recovery of patients [15]. TAP block is considered efficient in decreasing the requirement of pain-relief medication compared with WI. Other studies have also shown that TAP also reduces postoperative requirements of opiates [16].

A study was conducted by Petersen et al. to determine the beneficial impacts of TAP block after laparoscopic cholecystectomy in day-case surgery. The study found that patients who received TAP block after surgery had reported less coughing, lower pain scores along with decreased consumption of morphine. However, these reductions were small. The procedure has no reported complications and might be used as part of a multimodal analgesic treatment plan for day-case surgeries [17]. Khan et al. assessed ultrasound-guided TAP block efficacy in relieving pain post-surgery among patients undergoing lower abdominal surgery. The study found that TAP block is an effective mode of analgesia in the immediate and intraoperative postoperative period for patients undergoing inguinal hernia surgery and open appendectomy [18].

No TAP block-related consequences were identified in the current study; nevertheless, block failure, vascular injury, nerve injuries, and abdominal visceral are recognized as TAP block-related complications. TAP is better identified with ultrasound guidance, unproven needle control, and drug deposition is well guided under imaging. As a result, there were fewer problems and more clinically significant outcomes.

The current study determined pain score up to 6 hours after surgery. In the future, more trials need to be conducted to determine the long-term pain-relief effect of TAP block and WI. Second, this study was conducted only in one tertiary care hospital. In the future, more hospitals need to be involved in getting evident findings that can be incorporated into the practice setting.

## Conclusions

Compared to local anesthetic WI, ultrasound-guided TAP block has been demonstrated to be an effective method for providing appropriate postoperative analgesia among adult patients undergoing hernia repair in daycare procedures. However, more studies need to be conducted in the future, including large sample size and multiple centers, to get more generalizable findings.

## References

[1] Schug SA (2011). 2011--the global year against acute pain. Anaesth Intensive Care.

[2] Liu SS, Wu CL (2007). Effect of postoperative analgesia on major postoperative complications: a systematic update of the evidence. Anesth Analg.

[3] Edwards JE, McQuay HJ, Moore RA, Collins SL (1999). Reporting of adverse effects in clinical trials should be improved: lessons from acute postoperative pain. J Pain Symptom Manage.

[4] Coughlin SM, Karanicolas PJ, Emmerton-Coughlin HM, Kanbur B, Kanbur S, Colquhoun PH (2010). Better late than never? Impact of local analgesia timing on postoperative pain in laparoscopic surgery: a systematic review and metaanalysis. Surg Endosc.

[5] Rafi AN (2001). Abdominal field block: a new approach via the lumbar triangle. Anaesthesia.

[6] Hebbard P, Fujiwara Y, Shibata Y, Royse C (2007). Ultrasound-guided transversus abdominis plane (TAP) block. Anaesth Intensive Care.

[7] Albrecht E, Kirkham KR, Endersby RV (2013). Ultrasound-guided transversus abdominis plane (TAP) block for laparoscopic gastric-bypass surgery: a prospective randomized controlled double-blinded trial. Obes Surg.

[8] Fayezizadeh M, Majumder A, Neupane R, Elliott HL, Novitsky YW (2016). Efficacy of transversus abdominis plane block with liposomal bupivacaine during open abdominal wall reconstruction. Am J Surg.

[9] Gupta A (2005). Local anaesthesia for pain relief after laparoscopic cholecystectomy—a systematic review. Best Pract Res Clin Anaesthesiol.

[10] Kuppuvelumani P, Jaradi H, Delilkan A (1993). Abdominal nerve blockade for postoperative analgesia after caesarean section. Asia Oceania J Obstet Gynaecol.

[11] Skjelsager A, Ruhnau B, Kistorp TK, Kridina I, Hvarness H, Mathiesen O, Dahl JB (2013). Transversus abdominis plane block or subcutaneous wound infiltration after open radical prostatectomy: a randomized study. Acta Anaesthesiol Scand.

[12] Mukhtar K (2009). Transversus abdominis plane block. J NYSORA.

[13] Ali L, Waseem M, Iqbal A (2018). Comparison of analgesic efficacy of transversus abdominis plane block with conventional local anesthetic wound infiltration. PAFMJ.

[14] Ismail S, Khan MR, Urooj S (2013). Use of transversus abdominis plane block as an anesthetic technique in a high risk patient for abdominal wall surgery. J Anaesthesiol Clin Pharmacol.

[15] Jørgensen H, Wetterslev J, Møiniche S, Dahl JB (2000). Epidural local anaesthetics versus opioid-based analgesic regimens on postoperative gastrointestinal paralysis, PONV and pain after abdominal surgery. Cochrane Database Syst Rev.

[16] Gupta A, Favaios S, Perniola A, Magnuson A, Berggren L (2011). A meta-analysis of the efficacy of wound catheters for post-operative pain management. Acta Anaesthesiol Scand.

[17] Petersen PL, Stjernholm P, Kristiansen VB (2012). The beneficial effect of transversus abdominis plane block after laparoscopic cholecystectomy in day-case surgery: a randomized clinical trial. Anesth Analg.

[18] Khan SM, Nawaz S, Delvi MB, Alzahrani T (2012). Intraoperative ultrasound guided transversus abdominis plane block in lower abdominal surgery. Int J Perioperative Ultrasound Appl Technol.

